This article has been retracted.

# Artificial Intelligence Technology-Based Medical Information Processing and Emergency First Aid Nursing Management

**DOI:** 10.1155/2022/8677118

**Published:** 2022-02-04

**Authors:** Qing Liu, Liping Yang, Qingrong Peng

**Affiliations:** Department of Emergency, The First People's Hospital of Lianyungang, Lianyungang City, 222002, China

## Abstract

This study was aimed at exploring the new management mode of medical information processing and emergency first aid nursing management under the new artificial intelligence technology. This study will use the artificial intelligence algorithm to optimize medical information processing and emergency first aid nursing management process, in order to improve the efficiency of emergency department and first aid efficiency. The successful rescue rates of hemorrhagic shock, coma, dyspnea, and more than three organs injury were 96.7%, 92.5%, 93.7%, and 87.2%, respectively, after the emergency first aid nursing mode was used in the hospital emergency center. The success rates of first aid within three years were compared, which were 91.8%, 93.4%, and 94.2%, respectively, showing an increasing trend year by year. 255 emergency patients in five batches in June and five batches in July were selected as the research objects by convenience sampling method. Among them, 116 cases in June were taken as the experimental group, and 139 cases in July were taken as the control group, which was used to verify the efficiency of the design model in this study. The results showed that the triage time of the two groups was 8.16 ± 2.07 min and 19.21 ± 6.36 min, respectively, and the difference was statistically significant (*P* < 0.01). The triage coincidence rates were 96.35% and 90.04%, respectively, and the difference was statistically significant (*P* < 0.05). The research proved that the design of intelligent medical information processing and emergency first aid nursing management research model can effectively improve the triage efficiency of the wounded, assist the efficiency of emergency nursing of medical staff, and improve the survival rate of emergency patients, which is worthy of clinical promotion.

## 1. Introduction

Emergency treatment is an important consulting room independent of other departments of the hospital. It undertakes the emergency diagnosis and treatment of all diseases, regardless of the patient's individual situation, and regardless of time and place. It is important to ensure the safety of people's lives [1]. According to relevant incomplete statistics, the total number of emergency patients in China's top 100 hospitals in 2019 was 351 million, accounting for one-tenth of the total number of 34,354 registered hospitals, that is, in 2019, the number of emergency patients in national registered hospitals reached 3.5 billion, and the data showed an increasing trend year by year [2]. The majority of first aid can save lives if people are effectively treated within 10 minutes to one hour. Therefore, effective diversion and diagnosis and treatment optimization of emergency patients are inevitable requirement for the development of emergency department [3–5].

With the popularization and development of artificial intelligence technology, there are more choices for the processing of traditional Chinese medicine information in the medical system [6]. Because there are many critical patients in the emergency department and the number of patients is not fixed, a large number of critical patients often need first aid at the same time in a short time. Therefore, how to ensure the effective transmission of each medical information, the seamless connection of each medical link, and the effective treatment for each patient in the case of short time, large number of people, urgent tasks, busy turnover, and insufficient manpower are the top priority to save the lives of patients [7]. Therefore, it is an effective way to improve the work efficiency of the emergency department, reduce the workload of emergency medical staff, and improve the success rate of treatment of critically ill patients by integrated design of the whole emergency treatment, medical information circulation, patient diversion, and department turnover in advance and optimization by using artificial intelligence [8–10].

In emergency first aid nursing management process, it will be divided into many links and each link is closely linked [11]. First, from the 120 ambulances, preliminary first aid including hemostasis, cardiopulmonary resuscitation, and bone reduction will be carried out for patients. At the same time, the clinical signs and disease conditions of patients will also be preliminarily diagnosed through the on-board medical system. After the ambulance is escorted to the hospital, rapid clinical diagnosis and triage will be carried out, and the patients are divided and classified by triage, so that patients can get corresponding professional medical rescue. At the end of first aid, it is necessary to refer patients who are in need, and some patients need hospitalization nursing. At this time, the first aid medical information needs to be transferred in multiple departments [12–15]. Complete emergency first aid nursing management needs to cover the above aspects, complete medical information processing, and emergency first aid nursing management through medical staff, which not only provides a lot of meaningless repetitive work but also is difficult to avoid mistakes [16, 17].

Therefore, this study will use the Internet, 4G communication, local area network, and other information technologies to build a set of medical information processing and emergency first aid nursing management system based on artificial intelligence, and it was successfully applied to clinical emergency activities. The system realizes the information sharing between hospital emergency and medical staff in other departments, optimizes the transmission channel of medical information, and can play a scientific and effective shunt for patients, shorten the first aid time of individual patients, and effectively improve the success rate of patient treatment. The process system is mainly divided into two parts, which are applied to the optimization of the overall emergency first aid nursing management process and the medical information processing module based on artificial intelligence technology.

In summary, this study selects the emergency data in hospital within one year based on artificial intelligence medical information processing and emergency first aid nursing management system constructed in this study and randomly selects 10 batches of emergency patients admitted in the second year as the research object to study the reception efficiency of routine emergency process and emergency process constructed in this study.

## 2. Materials and Methods

### 2.1. Research Objects

In this study, 321 patients who were critically ill admitted to the hospital within one year were selected as the research subjects, including 83 cases of traffic accident injury. 125 cases were admitted because of sudden heart disease, stroke, shock, and other sudden diseases. 59 patients were admitted because of fighting, falling injury, and accidents. 17 cases were hospitalized because of food poisoning and misuse of toxic substances. The remaining inconvenience classification or too low number of patients was 37 cases. There were 196 males and 125 females. They were 5-78 years old with an average age of 35.5 ± 12.6 years old. According to the general emergency classification, 42 cases were grade I, 84 cases were grade II, 113 cases were grade III, and 82 cases were grade IV [18].

10 batches of 255 emergency patients admitted due to traffic accidents were selected by convenience sampling method in all patients in the second year. Among them, 116 patients in five batches in June were selected as the experimental group, including 83 males and 33 females, aged from 16 to 69 years with an average age of 24.7 ± 16.1 years. The maximum number of hospitalized patients in a single batch was 18, and the minimum number of hospitalized patients in a single batch was 2. In addition, 139 patients in five batches in July were selected as the control group, including 88 males and 51 females, aged from 16 to 71 years old, with an average age of 25.2 ± 18.4 years old. The maximum number of hospitalized patients in a single batch was 24, and the minimum number of hospitalized patients in a single batch was 2. This study had been approved by ethics committee of hospital, and patients' families had been informed of this study and signed informed consents.

There was no significant difference in the general clinical data between the two groups (*P* > 0.05), and the specific results are shown in Figure 1. Inclusion criteria include (1) age > 16 years old and (2) emergency patients caused by traffic accidents and accidents. Exclusion criteria include (1) emergency patients without trauma and (2) no other major fatal complications occurred.

### 2.2. Emergency First Aid Nursing Management System Process

The emergency first aid nursing management system process is shown in Figure 2.

In view of the emergency first aid nursing management and the construction of hospital information system, the emergency rescue process is roughly divided into three parts. The first part is “120 pre-hospital emergency.” By using 4G communication technology and even the latest 5G communication technology, the “120” emergency vehicle is connected with the internal and external network servers. The monitoring instruments in the vehicle are wirelessly communicated with high-speed data, so that the information such as vehicle condition, vehicle GPS, vehicle rescue monitoring video, patient signs data, patient ECG, and patient oxygen saturation are related to the emergency command center and emergency database. The relevant information data are transmitted in real time, which is convenient for information sharing and data archiving. The emergency management is moved forward to prepare for hospital emergency first aid nursing management. The second part is the emergency first aid nursing management in hospital. The workstations of department directors, doctors, and nurses in the hospital are associated with the triage workstation in the emergency department to facilitate hospital consultation. The third part is the management of hospital data. By transferring prehospital transmission information data and hospital emergency medical information to the hospital intranet and carrying out classified management, it is convenient for future use at any time.

### 2.3. Emergency Department Workstation System

As the forefront of emergency first aid work, an emergency workstation directly determines the efficiency of emergency first aid work and the effective rate of first aid, which is extremely important for the entire emergency department. By combining the rapid development of artificial intelligence technology with emergency diagnosis and treatment, a medical information processing system with emergency characteristics is constructed to greatly improve the efficiency of emergency first aid. In this study, based on the neural network algorithm, semantic network, natural language processing (NLP) algorithm, and the national diagnosis and treatment guidelines and related literature as data resources, it builds a set of medical information processing system based on ontology semantic medical knowledge base and AI reasoning engine as the core [19–22]. The system will follow the national clinical diagnosis and treatment norms, through big data to simulate the emergency first aid nursing management of clinicians, compare the input patient information with the database information, and provide all patients with auxiliary management including inquiry (for conscious patients), examination, diagnosis, and treatment. According to the characteristics of the emergency department, a supporting triage and preexamination system is also provided. Through database comparison and national clinical diagnosis and treatment norms, the emergency order of patients is arranged according to the critical grade of emergency nursing, and the patients with acute and critical diseases are given priority to as much as possible. The specific process is shown in Figure 3.

With the above management system, patients will be distinguished by identification wristbands. Three-color wristbands will be used for management according to patients' disease conditions. As shown in Figure 3, red, yellow, and green wristbands will be used. Red represents grade I and II patients, respectively, endangered patients and critically ill patients. Yellow is grade III, representing emergency patients. Green is a class IV patient, a nonemergency patient. Among them, red patients as key patients will have the highest priority for rescue, yellow patients as emergency patients will be treated as severe emergency, and green patients are ranked as the lowest priority in emergency first aid nursing management. The wristband will not only serve as the identification of triage sorting but also carry patient information and two-dimensional code, which will be used as the patient's personal information code for referral, registration, recharge and payment, printing laboratory sheet, fee inquiry, and other purposes.

The system will be connected to the “120” emergency vehicle intelligent system, the emergency department medical staff will receive the patient's medical information according to 4G or 5G communication technology, as early as possible to prepare for emergency. The patient's general personal information and specific medical information are compared and summarized when the patient reaches the emergency department, and the patient's information is professionally evaluated by the intelligent emergency workstation to assist the medical staff. For patients with high scores, the system will remind medical staff to be ready to contact specialists and be ready for referral as soon as possible. For emergency patients, the system will be connected with each bed monitor, ventilator, and other instruments, real-time collection of patients' medical information and file collection, and the patient's every link of information are concentrated in electronic files, in order to be convenient access at any time.

### 2.4. Effect Verification of Artificial Intelligence Emergency First Aid System

In order to verify the practical effectiveness of the artificial intelligence-based integrated medical information processing and emergency first aid nursing management system designed in this study, the experiment is divided into two parts. The first part is the verification of the intelligent emergency triage management system. This experiment uses the system in the emergency department for one year to collect the emergency response efficiency of various types of common emergency symptoms in this year, so as to observe the macroresponse efficiency of the emergency response nursing management system based on artificial intelligence. In the second part, a convenience sampling method will be used to select 10 batches of emergency patients treated as research objects; they are randomly divided into the experimental group and control group. The experimental group will use the artificial intelligence-based emergency first aid nursing management system designed in this study for first aid activities, while the control group will use the traditional manual receiving and triage method for first aid, so as to observe the triage time and triage coincidence rate of the system.

### 2.5. Evaluation Indicators

In this study, the average triage time, the coincidence rate of triage results, and the triage time of critically ill patients were compared between the two groups, which were used as the evaluation standard for the effective management of emergency care.

The average triage time refers to the time taken by patients from the triage station to the triage station. The triage time of critically ill patients refers to the definition of critically ill patients with CRAMS (Circulation, Respiration, Abdomen, Motor, Speech) trauma score ≤ 6 and modified early warning score (MEWS) ≥ 5. The coincidence rate of triage: in the two groups of patients, the random number table method was used to randomly extract the preexamination triage information of patients, and the triage level was hidden. Experts were invited to retrospectively triage, and the differences between the two triage levels were compared. The specific calculation formula is as follows.

(1) $$\begin{array}{c} T=\frac{A}{B}\times 100\%, \end{array}$$

where *T* is the coincidence rate of triage, *A* is the number of cases in which the retrospective triage results of experts are consistent with the original triage results, and *B* is the total number of patients extracted.

### 2.6. Statistical Method

The data in this study were analyzed by SPSS19.0 statistical software. The measurement data were expressed as mean ± standard deviation ($\overset{¯}{x}\pm s$), and the count data were expressed as percentage (%). One-way analysis of variance was used for pairwise comparison. *P* < 0.05 or *P* < 0.01 indicated that the difference was statistically significant.

## 3. Results

### 3.1. Integrated Medical Information Processing and Emergency First Aid Nursing Management Process Based on Artificial Intelligence

The following chart is the construction process of the integrated medical information processing and emergency first aid nursing management system based on artificial intelligence (Figure 4).

### 3.2. Rescue Results of Patients with Different Degrees of Illness

The types of diseases and the rescue success rate of severe traumatic complications in the emergency department within one year were summarized (Figures 5 and 6), and the first aid results within three years were compared (Figure 7).

Figure 5 is the type and proportion of common complications in emergency trauma patients within one year. According to Figures 6 and 7 data, it can be clearly reflected in the use of artificial intelligence-based integrated medical information processing and emergency first aid nursing management, the overall emergency first aid efficiency has gradually improved, and there is an obvious upward trend in three years.

### 3.3. Comparison of Emergency Effective Rate of Selected Patients

Figure 8 is the comparison of emergency triage time and emergency triage coincidence rate between the two groups. Triage time of the experimental group and the control group were 8.16 ± 2.07 min and 19.21 ± 6.36 min, respectively, and the difference was statistically significant (*P* < 0.01). The triage coincidence rates were 96.35% and 90.04%, respectively, and the difference was statistically significant (*P* < 0.05).

## 4. Discussion

At present, in the general emergency room triage, nurses perform emergency grade assessment according to the physician on the patient's self-report, clinical signs, disease performance, test data, and various scales of, and then, patients are divided into different grades. All medical accidents in Shanghai, China from 1990 to 2015 were statistically studied by Gao et al. [23]. The study found that the difference in diagnosis was the main error type in all medical accidents, and it mainly occurred in men, in the age group under 10 and 50-70 years old. Patients carrying respiratory diseases, tumors, and hypertension were independent predictors of error diagnosis. The conclusion showed clinical decision-making system can effectively improve the accuracy of clinical diagnosis in 68% of the experiments. Through research at home and abroad, the use of artificial intelligence technology to assist the medical room effectively reduces the effective means of medical accidents. The emergency department often appears a large number of critically ill patients need to be diagnosed at the same time, which causes great pressure on the medical staff of the emergency department, and often inevitably leads to misdiagnosis and missed diagnosis, resulting in aggravation, delay, and even death of critically ill patients. Therefore, it is an inevitable trend to introduce artificial intelligence technology into the emergency department.

This study is also based on the above reasons, through artificial intelligence technology for emergency medical information unified processing, and emergency first aid nursing management process optimization, in order to improve the efficiency of emergency first aid. This study innovatively introduces artificial intelligence, has a certain planning for the overall emergency first aid process, making hardware and software match each other, and has more efficient improvement efficiency. Through many years of clinical practice and extraction control experiment in the hospital, this study studies in detail the design of integrated medical information processing and emergency first aid nursing management system based on artificial intelligence in emergency first aid effectiveness and the speed and accuracy of triage. In the hospital emergency common complications, the rescue success rate of hemorrhagic shock was 96.7%, the rescue success rate of coma was 92.5%, the rescue success rate of dyspnea was 93.7%, and the rescue success rate of organ injury combined with more than three was 87.2%. The success rates of first aid in three years were compared, which were 91.8%, 93.4%, and 94.2%, respectively, showing an increasing trend year by year. The triage time of emergency patients with the system designed in this study was 8.16 ± 2.07 min, and the triage time of emergency patients with traditional emergency rescue process was 19.21 ± 6.36 min; the difference was statistically significant (*P* < 0.01). The triage coincidence rate of emergency patients using the system designed in this study was 96.35%, while that of emergency patients using the traditional emergency rescue process was 90.04%, and the difference was statistically significant (*P* < 0.05). As for Kawamoto et al. [24], through the application of clinical decision-making system in clinical practice, more than 70 related experimental reports were studied in multiple control test retrieval libraries. It is consistent with the results of this study. In summary, under the new management mode of medical information processing and emergency first aid nursing management under the new artificial intelligence technology, the triage efficiency of the wounded has been improved, the emergency nursing efficiency of auxiliary medical staff, and the survival rate of emergency patients have been improved.

## 5. Conclusion

In this study, the clinical data of three years of emergency treatment in the hospital were selected, and 10 batches of emergency patients were selected for emergency triage time and triage accuracy to study the integrated medical information processing and emergency first aid nursing management system based on artificial intelligence designed in this study. The results proved that the system can effectively improve the efficiency and accuracy of emergency first aid. There is the room for improvement in the construction of the system in this experiment. Especially, artificial intelligence should be more applied. It is expected that more domestic and foreign research can improve the research of artificial intelligence in the treatment and diagnosis. This study can play a guiding role in the improvement and construction of hospital emergency department and provide some experimental data.

## Figures and Tables

**Figure 1:** Comparison of individual clinical data of patients. Note: (a) The results of gender and age comparison between the two groups. (b) The comparison results of admission and emergency grading between the two groups.

**Figure 2:** General process of emergency first aid nursing management system.

**Figure 3:** Intelligent emergency triage management system.

**Figure 4:** Detailed process of emergency first aid nursing management ((a) the prehospital emergency part, (b) the emergency department workstation, (c) the command center, (d) the rescue area, and (e) the database).

**Figure 5:** Types of severe trauma complications.

**Figure 6:** Emergency effective rate of different complications.

**Figure 7:** Comparison of effective rate of emergency care in three years.

**Figure 8:** Comparison of triage time and coincidence rate between the two groups ((a) the proportion of emergency triage time in the two groups and (b) comparison of triage coincidence rate two groups; in (a), compared with the experimental group, $\overset{*}{\;\;}P$ <0.01; in (b), compared with the experimental group, ^*P* < 0.05).

## Data Availability

The data used to support the findings of this study are available from the corresponding author upon request.
